The article "Optimization of Precious Metals Recovery from Electronic Waste by Chromobacterium violaceum Using Response Surface Methodology (RSM)" was published in 2023. Journal: Bioinorg Chem Appl.

# Optimization of Precious Metals Recovery from Electronic Waste by *Chromobacterium violaceum* Using Response Surface Methodology (RSM)

**DOI:** 10.1155/2023/4011670

**Published:** 2023-03-30

**Authors:** Wan Nur Fazlina Abdol Jani, Fatihah Suja', Sharifah Iziuna Sayed Jamaludin, Nor Fadilah Mohamad, Noor Hidayu Abdul Rani

**Affiliations:** ^1^School of Chemical Engineering, College of Engineering, Universiti Teknologi MARA Johor Branch, Pasir Gudang Campus, 81750 Bandar Seri Alam, Masai, Johor, Malaysia; ^2^Department of Civil & Structural Engineering, Faculty of Engineering & Built Environment, Universiti Kebangsaan Malaysia, Bangi 43600, Selangor, Malaysia

## Abstract

An effective recovery technology will be valuable in the future because the concentration of the precious metal contained in the source can be a key driver in recycling technology. This study aims to use response surface methodology (RSM) through Minitab software to discover the optimum oxygen level (mgL^−1^), e-waste pulp density (% w/v), and glycine concentration (mgL^−1^) for the maximum recovery of gold (Au) and silver (Ag). The method of precious metals recovery used for this study was taken from the bioleaching using 2 L of batch stirred tank reactor (BSTR). A Box-Behnken of RSM experimental statistical designs was used to optimize the experimental procedure. The result of the RSM optimization showed that the highest recovery was achieved at an oxygen concentration of 0.56 mgL^−1^, a pulp density of 1.95%, and a glycine concentration of 2.49 mgL^−1^, which resulted in the recovery of 62.40% of Au. The pulp density and glycine concentration greatly impact how much Au is bioleached by *C. violaceum*. As a result, not all of the variables analyzed seem crucial for getting the best precious metals recovery, and some adjustments may be useful in the future.

## 1. Introduction

In the present world, having electronic devices has become a need. These devices are essential for human communication and daily convenience. Up to 60 different metals can be found in modern electronics, and to make up for any potential shortage, there is a growing interest in secondary sources of these metals, particularly e-waste [1]. According to the European Union (EU) directive, e-waste is any waste of electrical and electronic equipment, including all components, subassembly, and consumables, or any part of the discarded product deemed unnecessary [2]. E-waste contains more than 1000 components, hazardous materials—cadmium (Cd), chromium (Cr), lead (Pb), and mercury (Hg)—and nonferrous metals such as aluminium (Al) and copper (Cu). In addition to base metals, e-waste, e.g., PCBs, also contains precious metals, such as gold (Au), silver (Ag), and platinum (Pt) [3]. Due to their high chemical stability and excellent conducting qualities, these metals are frequently used in the production of electrical products [4]. Although PCBs concentrations are not as high as base metals, this valuable resource is more difficult to find in original compounds on the Earth. Surprisingly, the concentrations of precious metals in PCBs can be more than ten times greater than those of commercially mined minerals [5]. An electronic device includes a component primarily made of toxic metals and chemicals. Such materials include beryllium (Be), phthalates, polyvinyl chloride (PVC), brominated flame retardants (BFRs), and antimony [6, 7]. A significant reason for the rapid generation of e-waste is the high rate of obsolescence in the electronic market, particularly in developing countries [8]. Most electronic products are changed at least every two years, have a relatively short shelf life, and are either abandoned or exported as used goods to underdeveloped nations.

Environmental pollution has resulted from the breakdown and disposal of e-waste. According to data provided by Jaibee et al. [7]; landfills have received more than 90% of unnecessary electrical and electronic waste. As a result, landfills are producing an increasing amount of e-waste, worsening the degradation of the environment. Cancer risk increases along with developmental and neurological issues [9]. Additionally, incinerating has harmed the environment, particularly in the quality of solids, land, and air. When computer chip sludge and acid are dumped on the ground, the soil becomes more acidic, contaminating water sources [10]. Even worse, past research has revealed some health issues brought on by the hazardous metal and chemical effects of e-waste. A review conducted by Pant [11] confirmed the toxic effects of metals such as Pb, Cd, Hg, Cr, arsenic (As), nickel (Ni), selenium (Se), lithium (Li), and americium (Am) on the human body.

Microorganisms, particularly cyanogenic bacteria, have come under consideration as a potential alternative method for the gold cyanidation process in recent years. Microbes such as *A. ferrooxidans*, *C. violaceum*, and *Aspergillus* sp. increased gold and Cu recovery from e-waste, especially mobile-PCBs [12–14]. It has long been known that aerobic gram-negative bacteria can produce free cyanide [15], which Sneath and Punjab [16] initially discovered in mesophilic *C. violaceum* strains. *C. violaceum* is a mesophilic, motile, gram-negative, and facultative anaerobe [17]. This bacterial strain exhibits excellent potential for the ecological gold recovery technique [18, 19]. Several physiological and nutritional factors (pH, temperature, glycine concentration, pulp density, and medium composition) may affect the process's end product [20]. Therefore, process optimization is needed to achieve maximal recovery with the fewest number of experiments. In this situation, statistical techniques can identify interactions between factors. The response surface methodology (RSM) has been used to model, evaluate, and research the relationship and interaction of the individual components [21]. Only a few studies have been done using RSM for bioleaching metals from e-waste [22].

The recovery of Au and Ag metals from e-waste is widely studied in this research. E-waste mobile-PCBs were converted into ingots and leached using the batch stirred tank reactor (BSTR) technique. The experimental findings are verified using RSM software for various factors, including oxygen level, e-waste pulp density % (w/v), and glycine concentration.

## 2. Materials and Methods

### 2.1. Source of Mobile-PCBs Concentrates

The e-waste focusing on mobile-PCBs is sourced from a local electronic mobile shop in Selangor, Malaysia. No physical and mechanical methods are applied to the sample before it is transported to the laboratory to avoid the loss of its properties. The scrap mobile-PCBs (SW110) is first manually crushed to a uniformity of 500 *μ*m using stainless steel scissor. The analysis is then performed using the representative samples. Then, 100 mL of aqua regia solution, 68% concentrated HNO_3_, and 37% concentrated HCl (HNO_3_ : HCl = 1 : 3), is used to dissolve 1 g of mobile-PCBs [23]. The solution is refluxed in a 250 mL beaker for 1 hour at 100°C. After the solution cools, the volume of solution is made up to 100 mL with deionised water. Then, the solution is passed through glass fibre filters (PALL-GF-A/E-1) to guarantee particle-free suspensions and stored at 4°C for further analysis. Next, the mobile-PCB undergoes an inductively coupled plasma-mass spectrometry (ICP-MS) (Brand Perkin Elmer, Model NEXION 2000) technique to identify the metal content in the metal concentrates. The APHA Method 6020B ICP-MS analysis was used to conduct the procedure, which involved inserting a sample of filtered effluent into the ICP-MS apparatus. 15 mL of pure mobile-PCBs after the aqua regia leaching was used to determine the Au and Ag concentration using ICP-MS testing. The fine mobile-PCBs (of particle size less than 1.0 mm) are then sterilised via autoclaving at 121°C for 15 minutes for the bioleaching study [24].

E-waste may contain harmful contaminants if mismanaged. The first step in the isolation and purification process employed throughout the research was the manual physical separation of various forms of e-waste into distinct categories such as metals, plastics, and glass. Next, precious metals are extracted from e-waste via a bioleaching method utilising *C. violaceum*. Finally, impurities that cannot be purified must be properly disposed of to protect the environment and public health.

### 2.2. Single-Culture Cyanogenic Bacteria

The bacteria used in this study are single-culture cyanogenic bacteria, namely, *C. violaceum* (strain DSMZ 30191). These bacteria are purchased from the German Collection of Microorganisms and Cell Culture (DSMZ), Braunschweig, Germany, in an actively growing culture (agar slant). Prior to its adaptation in this study, the *C. violaceum* must undergo at least twice-duplicate subculturing to prove its authenticity, which is done through identification techniques. The *C. violaceum* is inoculated from single colonies of one loop full of slant in both nutrient agar (BD 213000) and nutrient broth (BD 234000) media for 24 hours under a stationary phase at 30°C. After an overnight confluent culture, isolated organisms are characterised according to basic morphological techniques, including morphology (classified via size, shape, appearance, and colour), gram staining reaction count, and turbidity measurement through optical density determination. After completion of the identification techniques, the *C. violaceum* is subcultured in LB broth (Difco) under a stationary phase at 30°C, and transferred twice a month. Long-term storage of the organism is held in 2 mL cryotubes with 500 *μ*L of 20% glycerol, and 500 *μ*L of liquid inoculated medium at −20°C.

To obtain the optimum free cyanide formation by *C. violaceum*, the media used are Luria Bertani broth (LB) comprising (in gL^−1^) of 10 tryptone, 5 yeast extract, 0.75 glycine, and 10 NaCl. All media are autoclaved at 121°C for 15 minutes and cooled to room temperature before being transferred into a 2.5 L batch stirred tank reactor (BSTR) for the bioleaching study. The dissolution of Au in cyanide solution consists of anodic and cathodic reactions as stated in the Elsner's equations by J.A. Cook [25]:

(1) $$\begin{array}{c} 4Au+8{CN}^{-}⟶4Au{\left(CN\right)}_{2^{-}}+4e^{-} \end{array}$$

(2) $$\begin{array}{c} O_{2}+2H_{2}O+4e^{-}⟶4{OH}^{-} \end{array}$$

(3) $$\begin{array}{c} 4Au+8{CN}^{-}+O_{2}+2H_{2}O⟶4Au{\left(CN\right)}_{2^{-}}+4{OH}^{-}\text{.} \end{array}$$

### 2.3. Bioleaching Process

A 2.5 L BSTR is used in experiments on the two-step bioleaching of mobile-PCBs. The acrylic fibre tank used by the BSTR tank has a 2.5 L tank volume (at a height/diameter ratio of 2.0). A mechanical stirrer that penetrates the tank at a 45-degree angle is present. The BSTR system was designed with a height of 27 cm and an internal diameter of 13 cm in downward aerobic flow (without recycling). The bioreactor's top provides access to the medium and mobile-PCB feeds. Daily output samples are collected through a sampling valve built 25 cm below the bioreactor's top. The waste the bioreactor has processed will be used as an effluent product, which will take the form of an ingot solution. To investigate the impact of aeration on the dissolution of precious metals using the BSTR method, pure air was supplied at a flowrate of 0.5 Lmin^−1^ and was produced by a gas compressor. In contrast, the gas compressor was turned off throughout the BSTR procedure at the nonaerated state (0.0 Lmin^−1^). During the 14-day incubation period, no controls were utilised to regulate the reactor's temperature or pH.  Figure 1 displays BSTR employed in the study. In earlier investigations, two-step bioleaching (indirect bacterial leaching) was preferred over direct bacterial leaching. This is such that even if microorganisms do not directly interact with the minerals, they do oxidise the ores through the leaching agents they produce [3].

Additionally, it was thought that the two-step procedure would boost metal mobilisation yield and decrease lixiviant usage [1]. First, 2 L of a sterile medium with a pH of 7.0 is added by inoculating it with a single culture of *C. violaceum* at a rate of 5% v/v. A gas compressor concurrently supplies pure air. 1% (w/v) pulp density of mobile-PCB was applied under aseptic circumstances after two days of incubation. It is known that different amounts of metals can be separated depending on the organism and the growth conditions used. Selection of the right microorganisms, i.e., acidophilic or alkalophilic in terms of cyanogenic types of bacteria, has produced efficient metal bioleaching techniques. The physical stability of isolated metals can be confirmed through the ability of ingots solution to detect the AuCN_2_^−^ solution (chemical formula for gold cyanide anion) at higher concentration, observe its color change over the bioleaching process, as well as the ability of *C. violaceum* to react well in 14-dat incubation period. Following a 14-day incubation period, a BSTR containing *C. violaceum* inoculum, medium, and mobile-PCBs was operated to provide the best output (when the observed yield difference was less than 5%).

45 mL of yield samples were drawn from the BSTR sampling output valve every two days and examined. Free cyanide concentration (CN^−^) was measured using a cyanide test kit quantofix technique (macherey-Nagel GMbH & CO. KG) and pH was determined using a YSI 556 pH metre. A DR 6000 HACH spectrophotometer was used to measure the optical density (OD) at a wavelength of 600 nm. The experiment was conducted by measuring the absorbance of each sample using a 3 mL disposable cuvette, and a blank sample of LB medium without *C. violaceum* was used as a control. These parameters' findings are indicated in units Abs. This procedure is carried out in accordance with the standard method OD in microbiology (OD600). 15 mL of pure mobile-PCBs after the bioleaching were then examined for the concentration of the metal ions Au and Ag using an ICP-MS apparatus after being filtered through a membrane nitrocellulose filter to ensure a suspension free of particles.

### 2.4. RSM Analysis

Design of experiment (DOE) is a useful approach that may be applied in various experimental contexts [26]. By connecting the quantitative data from experiments to mathematical and statistical equations, the design of experiment (DOE) modeling technique known as RSM can determine the relative impact of parameter variation and make parameter optimization easier [27].

Three factors, including e-waste pulp density, oxygen level and additive (glycine) concentration, were optimized by box-Behnken RSM using the Minitab version 20 software to achieve maximum Au and Ag recovery. The recovery of precious metals was taken as the RSM system's response. The quadratic equation model predicting the optimal point was expressed according to the following equation:

(4) $$\begin{array}{c} y=\beta 0+\overset{k}{\underset{i=1}{\sum }}\beta iXi+\overset{k}{\underset{i=1}{\sum }}\beta iiXi2+\overset{k-1}{\underset{i=1}{\sum }}\overset{k}{\underset{j=2}{\sum }}\beta ijXiXj+\varepsilon \text{,} \end{array}$$

where *y* is the response variable, *x*_*i*_ and *x*_*j*_ are coded independent variables, *β*_0_, *β*_*i*_, *β*_*ii*_, *β*_*ij*_ (*i* = 1, 2,…, *k*), and *β*_*ij*_ (*i* = 1, 2,…, *k*; *j* = 1, 2,…, *k*) are regression coefficients for intercept, linear, quadratic, and interaction terms, respectively, and *ε* is the statistical error. This equation represents an empirical relationship between the yield and the independent parameter obtained from response surface methodology modeling by the Box-Behnken (regression equation) method. RSM is a method for predicting and modeling complex relationships between independent variables and one or more responses [27].

Each variable has three coding levels: low (−1), middle (0), and high (+1). To examine the pure error at the design centre, 15 run trials with three components were conducted. The cubic model was used to select this optimization (Box-Behnken).  Table 1 displays the experimental design's list of variables and their respective levels.

## 3. Results and Discussion

### 3.1. Characterization of Mobile-PCBs

The results of the metal content of mobile-PCBs are shown in Table 2 and were previously reported in our study [28]. The amount of Cu (30.07 ± 0.200% w/w) was in the majority. The precious metals Au (0.01 ± 0.001%) and Ag (0.02 ± 0.005%) were in significantly lower quantities. The Au content in the mobile-PCBs is higher than that reported by Liang et al. [29] (0.004% Au) and comparable with electronic scrap materials (ESM) used by Tay et al. [30], i.e., 0.02% Au. Although the content of Cu was higher than that reported in Pradhan & Kumar [24], i.e., 12.06% Cu, the gold content was slightly lower (0.08% Au). The difference in metal contents, especially Au, is due to different e-waste sources (computer and scrap), influenced by the material's heterogeneity and origin.

### 3.2. RSM-Based Optimization

#### 3.2.1. Statistical Evaluation

The regression equation was used to determine the interaction between the three essential factors and precious metals recovery. Equations (5) and (6) shows the regression equation for the RSM data graphs for Au and Ag, respectively:

(5) $$\begin{array}{c} Au\;recovery\left(\%\right)=59.24+6.19X_{1}-9.90X_{2}-2.03X_{3}-34.35X_{1}*X_{1}-14.80X_{2}*X_{2}-17.33X_{3}*X_{3}-2.17X_{1}*X_{2}-0.96X_{1}*X_{3}+0.81X_{2}*X_{3}, \end{array}$$

(6) $$\begin{array}{c} Ag\;recovery\left(\%\right)=9.36+0.252X_{1}-1.620X_{2}+X_{3}-5.96X_{1}*X_{1}-3.17X_{2}*X_{2}-3.00X_{3}*X_{3}-0.15X_{1}*X_{2}-0.05X_{1}*X_{3}-2.71X_{2}*X_{3}\text{.} \end{array}$$

The Box-Behnken of RSM was used to optimize different factors (oxygen level, e-waste pulp density, and glycine concentration) affecting the recovery of metals during bioleaching. As a function of the independent factors, data on the dependent variables (oxygen level, e-waste pulp density, and glycine concentration) were fitted to a second-order equation (Equations (5) and (6)). The 15 experimental and predicted responses are presented in Table 3, and the statistical analysis of these data was performed at a confidence level of 95% (*P* < 0.05). The coefficient of determination (*R*^2^) measures the degree of fit and is defined as the ratio of the explained variance to the overall variation [31]. All the models had high precision (*R*^2^ near 1), indicating that the model explained the variability in the data.

Based on Table 3 results, the Au and Ag recovered in this study ranged from 1.81 to 59.24% and from 0.02 to 11.65%, respectively. The value of *R*^2^ in this recovery of Au and Ag is 0.956 and 0.885. To investigate the effect of each parameter on precious metals recovery, the analysis of variance (ANOVA) is shown in Table 4. ANOVA led to two modified quadratic models for both responses [22]. The *P* value from the coded coefficient table can be used to identify the component affecting precious metals recovery; the *P* value must be less than 0.05. Because *X*_2_ has a *P* value of 0.016, which is less than 0.05, it impacts the Au recovery. Next, the finding demonstrates that Ag recovery is influenced by *X*_1_*X*_1_. The lack-of-fit of the model is higher than 0.05 and is not significant, denoting that the model can fit experimental data with analytical data from the model.

#### 3.2.2. Response Plots

*(1) Au Recovery*. Au recovery was accomplished using a two-step bioleaching process and the BSTR technique. Biogenic cyanide interacts with gold during the two-step bioleaching process to generate the water-soluble complex dicyanoaurate [18]. Au leached out using *C. violaceum* under two-step bioleaching are comparable to the studies of [12, 24, 29], with 68.50, 69.30, and 70.60% w/w of Au being bioleached, respectively. On the other hand, the bioleach obtained was higher than those reported by Kita et al. [32]; Pham & Ting [33]; Tay et al. [30], Dangton and Leepowpanth [34] and Das et al. [35]; with a maximum of Au bioleachability, 60.00, 3.00, 30.00, 13.62, and 11.30% w/w, respectively. Instead of a batch reactor, shaking flasks were used in all prior research.

Figures 2(a)–2(c) show the relationship between Au recovery and these three parameters, the relationship of RSM will only focus on the e-waste pulp density (*X*_2_).  Figure 2(a) illustrates the interaction effect of oxygen level and e-waste pulp density on Au recovery. The maximum Au recovery was observed at the optimum pulp density of 2.75% (w/v), converging with the optimum oxygen level at 0.5 mgL^−1^. It was observed that increasing the pulp density above 2.75% reduced Au recovery. Environmental toxicity increases at higher e-waste pulp density, but bacterial activity decreases. Increasing pulp density would decrease the metal's recovery [33]. For instance, the leach solution must be prepared around the oxygen level's center point (0.5 mgL^−1^) and e-waste pulp density (2.75% w/v) to obtain a higher Au recovery. Besides that, Figure 2(c) represents the interaction effect of glycine concentration and e-waste pulp density on Au recovery. At a constant oxygen level of 0.5 mgL^−1^, the recovery of Au is represented by varying the glycine concentration from 0.75 to 4.50 mgL^−1^. While it also varies the pulp density from 0.5 to 5.0% (w/v). Increased glycine concentration from 2.2 to 3.0 mgL^−1^ increased Au recovery. However, due to the toxic effect of glycine on bacterial growth, the Au recovery decreased as the glycine concentration increased over 3.0 mgL^−1^.

*(2) Ag Recovery*. The result values in Table 3 will develop a response contour plot and surface plot for Ag recovery to facilitate seeing the best recovery results. Thus, in Figure 3, the response contour plot and surface plot for Ag recovery as a function of (a) oxygen level and e-waste pulp density is the best recovery for Ag. The darkest center can be represented as the highest value of Ag recovery on the contour plot. Furthermore, the parameters associated with this contour and surface plot are oxygen level and e-waste pulp density, where the value for oxygen level is 0.50 mgL^−1^ and 2.75 (% w/v) for e-waste pulp density. This means that the absence of glycine concentrations does not affect the recovery process to get the highest recovery for Ag. Combining two parameters alone can also obtain the highest recovery meaning that the perfect recovery needs to be mixed up oxygen level and e-waste pulp density.

#### 3.2.3. Process Optimization and Model Validation

Optimization of the variables was then identified using the response optimizer function in the Minitab software version 20. Figures 4 and 5 show the optimization results for Au and Ag recovery as a function of oxygen level (*X*_1_), e-waste pulp density (% w/v) (*X*_2_), and glycine concentration (*X*_3_), respectively. Then, to confirm the validity of the models, an independent bioleaching experiment using BSTR was performed under optimal conditions as prescribed by the software. Point prediction and experimental recovery of precious metals (Au and Ag) under optimal statistical conditions for model validation and accuracy was included in Table 5.

A maximum Au recovery desirability of 61.32% was predicted for the response variable targets with an oxygen level of 0.56 mgL^−1^, e-waste pulp density of 1.95% (w/v), and glycine concentration of 2.49 mg/L. It is worth noting that the optimized Au recovery is obtained by decreasing the total value of e-waste pulp density, previously used at 2.75% w/v. However, the predicted Ag recovery is still low, even using the variables under optimum conditions (with an oxygen level of 0.52 mgL^−1^, e-waste pulp density of 1.77% (w/v), and glycine concentration of 3.40 mg/L). The confirmatory results showed that the obtained responses for Au (62.40%) and Ag (10.33%) recovery agreed well with the predicted responses. Based on the experiment conducted on the Ag recovery from e-waste, it can be concluded that the experimental recovery value does not guarantee getting the highest predicted value. As a result, more parameters must be involved than just the three necessary ones in order to obtain the best finding. It is important to stress the study of pH, particle size, and the use of various microbes. pH is a general factor but greatly impacts the Au and Ag recovery process. E-waste has been reported to be alkaline, increasing the medium's pH. The dissolution of precious metals is very slow, below pH 6.8 or above pH 9.5 [36]. Then, the particle size of the e-waste source is also a factor in increasing the effectiveness of the 2-step bioleaching process. When generally solid e-waste is put into a liquid medium and reacts together, the particles between the two cannot combine, but only the particles on the surface of the e-waste will come into contact with the medium. Therefore, breaking the e-waste into small pieces, such a thing allows for an increase in the surface area ratio (area per total sample) and guarantees the activity of microorganisms to react in the dissolution of Au metal. Generally, a sieve fraction of 0.5 mm to 1.0 mm is selected for experimental research [37].

## 4. Conclusion

Two-step bioleaching process using BSTR was optimized to leach only Au metal from e-waste mobile-PCBs using Box-Behnken RSM by a cyanogenic bacterium *C. violaceum*. One quadratic model was proposed by RSM, which can be utilized as an efficient tool to predict Au recovery through bioleaching. The maximum recovery occurred at an oxygen level of 0.56 mgL^−1^, pulp density 1.95%, and glycine concentration 2.49 mgL^−1^, which led to the extraction of 62.40% of Au. The pulp density and glycine content greatly influence the bioleaching of Au by *C. violaceum*, as the recovery of the metal would be reduced by increasing pulp density. Glycine concentrations beyond 3.0 mgL^−1^ were associated with a reduction in Au recovery. However, under the optimal condition suggested by the Ag model, only 10.33% of Ag was extracted (at an oxygen level of 0.52 mgL^−1^, pulp density 1.77%, and glycine concentration 3.40 mgL^−1^). It can be inferred from the experiment on Ag recovery from e-waste that the experimental recovery value does not ensure receiving the greatest predicted value. Therefore, further investigation and improvement regarding parameters influencing metal bioleaching should be undertaken.

## Figures and Tables

**Figure 1:** BSTR used in a two-step bioleaching process.

**Figure 2:** Contour plot and surface plot for Au recovery as a function of (a) oxygen level and e-waste pulp density; (b) oxygen level and glycine concentration; and (c) e-waste pulp density and glycine concentration.

**Figure 3:** Contour plot and surface plot for Ag recovery as a function of (a) oxygen level and e-waste pulp density; (b) oxygen level and glycine concentration; and (c) e-waste pulp density and glycine concentration.

**Figure 4:** The optimization results for Au recovery as a function of oxygen level (*X*_1_), e-waste pulp density (% w/v) (*X*_2_), and glycine concentration (*X*_3_).

**Figure 5:** The optimization results for Ag recovery as a function of oxygen level (*X*_1_), e-waste pulp density (% w/v) (*X*_2_), and glycine concentration (*X*_3_).

**Table 1:** Levels and factors variables in the experimental design.

Factors	Variables	Units	Code levels		
			−1	0	+1
*X*_1_	Oxygen level	(mgL^−1^)	0.0	0.5	1.0
*X*_2_	E-waste pulp density	(%)	0.50	2.75	5.00
*X*_3_	Glycine concentration	(mgL^−1^)	0.750	2.625	4.500

**Table 2:** Composition of scrap mobile-PCBs.

Metals	Content % (w/w)
Copper, Cu	30.07 ± 0.200
Iron, Fe	9.07 ± 0.010
Chromium, Cr	2.59 ± 0.003
Selenium, Sn	2.40 ± 0.010
Zinc, Zn	1.97 ± 0.002
Silver, Ag	0.02 ± 0.005
Gold, Au	0.01 ± 0.001

**Table 3:** Experimental design with factors and level suggested by Box-Behnken RSM, along with experimental and predicted results.

Run order	Factors			Experimental				Predicted	
	*X*_1_	*X*_2_	*X*_3_	Au (mgL^−1^)	Ag (mgL^−1^)	Au (%)	Ag (%)	Au (%)	(Ag)
1	0.0	0.50	2.625	0.044	0.007	4.50	0.07	11.62	1.45
2	1.0	0.50	2.625	0.227	0.018	23.20	0.73	28.35	2.25
3	0.0	5.00	2.625	0.013	0.002	1.32	0.02	3.83	1.50
4	1.0	5.00	2.625	0.111	0.002	11.33	0.10	4.21	1.29
5	0.0	2.75	0.750	0.050	0.002	2.90	0.07	2.44	1.23
6	1.0	2.75	0.750	0.149	0.020	15.22	0.81	16.73	0.62
7	0.0	2.75	4.500	0.018	0.002	1.81	0.09	0.30	1.52
8	1.0	2.75	4.500	0.101	0.015	10.31	0.62	10.77	1.92
9	0.5	0.50	0.750	0.455	0.021	46.50	0.87	39.83	0.78
10	0.5	5.00	0.750	0.125	0.003	12.81	0.14	18.42	2.95
11	0.5	0.50	4.500	0.389	0.286	39.77	11.65	34.16	8.84
12	0.5	5.00	4.500	0.091	0.002	9.33	0.10	15.99	0.19
13	0.5	2.75	2.626	0.580	0.230	59.24	9.36	59.24	9.36
14	0.5	2.75	2.625	0.580	0.230	59.24	9.36	59.24	9.36
15	0.5	2.75	2.625	0.580	0.230	59.24	9.36	59.24	9.36

**Table 4:** ANOVA for quadratic model of Au and Ag (%) recovery.

Response	Source	Sum of squares	Df	Mean square	*F*-value	*P* value	95% CI
Au recovery (%)	Model	6767.03	9	751.89	12.08	0.007	
	*X*_1_-oxygen level	306.65	1	306.65	4.93	0.077	(0.29, 0.71)
	*X*_2_-pulp density	783.68	1	783.68	12.60	0.016	(1.81, 3.69)
	*X*_3_-glycine concentration	32.85	1	32.85	0.53	0.500	(1.84, 3.41)
	*X*_1_ *∗* *X*_1_	4356.00	1	4356.00	70.01	0.000	
	*X*_2_ *∗* *X*_2_	809.31	1	809.31	13.01	0.015	
	*X*_3_ *∗* *X*_3_	1109.23	1	1109.23	17.83	0.008	
	*X*_1_ *∗* *X*_2_	18.88	1	18.88	0.30	0.605	
	*X*_1_ *∗* *X*_3_	3.65	1	3.65	0.06	0.818	
	*X*_2_ *∗* *X*_3_	2.64	1	2.64	0.04	0.845	
	Error	311.10	5	62.22			
	Lack-of-fit	311.10	3	103.70	^*∗*^	^*∗*^	
	Pure error	0.000	2	0.000			
	Total	7078.14	14				
	*R* ^2^ = 0.956						
	Adjusted *R*^2^ = 0.8769						

Ag recovery (%)	Model	243.924	9	27.103	4.27	0.062	
	*X*_1_-oxygen level	0.505	1	0.505	0.08	0.789	(0.29, 0.71)
	*X*_2_-pulp density	20.995	1	20.995	3.31	0.129	(1.81, 3.69)
	*X*_3_-glycine concentration	13.966	1	13.966	2.20	0.198	(1.84, 3.41)
	*X*_1_ *∗* *X*_1_	131.212	1	131.212	20.67	0.006	
	*X*_2_ *∗* *X*_2_	37.074	1	37.074	5.84	0.060	
	*X*_3_ *∗* *X*_3_	33.258	1	33.258	5.24	0.071	
	*X*_1_ *∗* *X*_2_	0.084	1	0.084	0.01	0.913	
	*X*_1_ *∗* *X*_3_	0.011	1	0.011	0.00	0.968	
	*X*_2_ *∗* *X*_3_	29.268	1	29.268	4.61	0.085	
	Error	31.734	5	6.347			
	Lack-of-fit	31.374	3	10/578	^*∗*^	^*∗*^	
	Pure error	0.000	2	0.000			
	Total	275.658	14				
	*R* ^2^ = 0.885						
	Adjusted *R*^2^ = 0.6777						

^*∗*^Df, degree of freedom; CI, confidence interval.

**Table 5:** Point prediction and experimental recovery of precious metals (Au and Ag) under optimal statistical conditions for model validation and accuracy.

Response	*X*_1_, oxygen level (mgL^−1^)	*X*_2_, E-wastepulp density (%)	*X*_3_, glycine concentration (mgL^−1^)	Predicted response (%)	Actual response (%)
Au recovery	0.56	1.95	2.49	61.32	62.40
Ag recovery	0.52	1.77	3.40	9.99	10.33

## Data Availability

The results (Table 2) data used to support the findings of this study have been deposited in the Abdol Jani et al. [28] repository (SSRN: https://ssrn.com/abstract=4165436 or https://doi.org/10.2139/ssrn.4165436).
